# The Effect of Off-Pump Coronary Artery Bypass Grafting in Patients on Aspirin Therapy until Surgery Day

**DOI:** 10.1155/2022/8674401

**Published:** 2022-07-08

**Authors:** Zhishuo Liu, Zhonglu Yang, Yuguang Ge, Lu Wang, Hui Jiang

**Affiliations:** ^1^Department of Cardiovascular Surgery, HeBei PetroChina Central Hospital, Langfang 065000, China; ^2^Department of Cardiovascular Surgery, General Hospital of Northern Theatre Command, Shenyang 110000, China

## Abstract

Coronary artery bypass grafting (CABG) is widely used to treat coronary artery disease, and intraoperative and postoperative bleeding is one of the major factors affecting the efficacy and mortality of CABG. To overcome the adverse effects of extracorporeal circulation (CPB), nonextracorporeal coronary artery bypass grafting (OPCABG) has become the main modality of CABG but is still prone to thromboembolic events. Whether antiplatelet agents should be clinically applied before CABG, especially OPCABG, remains controversial. Aspirin is currently the most important perioperative oral antiplatelet agent for coronary artery bypass graft surgery. In this study, we evaluated the effect of continuing aspirin therapy before OPCABG and observed perioperative performance and physiological indicators to find evidence for continuing aspirin therapy before surgery in China. The study showed that preoperative aspirin application had a positive effect on enhancing early postoperative platelet inhibition without increasing the incidence of adverse effects such as cardiovascular events. This provides an important clinical reference for whether antiplatelet agents should be applied before CABG, especially OPCABG.

## 1. Introduction

Nowadays coronary artery bypass grafting (CABG) has been widely performed for coronary artery disease [1]. In order to overcome the adverse effect of cardiopulmonary bypass (CPB), off-pump coronary artery bypass grafting (OPCABG) has become the main way of CABG. OPCABG not only reduces surgical trauma but also reduces the impact on patients' coagulation function damage. Even so, intraoperative and postoperative bleeding is still one of the main factors that influence the efficacy of CABG and mortality, while OPCABG is an independent risk factor for thromboembolic events [2, 3]. For this reason, whether antiplatelet drugs should be applied clinically before CABG, especially OPCABG, is still under debate [4].

Aspirin is currently the most important perioperative oral antiplatelet drug for coronary artery bypass surgery. It irreversibly inactivates platelet cyclooxygenase (COX)-1 and acetylates the serine residue (Ser-529) in the polypeptide chain of the active site to inhibit the production of TXA2, thereby inhibiting platelets [5]. For patients undergoing OPCABG, some early reports suggest that patients should stop using antiplatelet drugs for 5–7 days before CABG surgery, which is still the theoretical basis for some cardiac surgeons to stop aspirin before surgery [6]. In some medical institutions, low-molecular-weight heparin was replaced for aspirin. With the deepening of research, some literature reported application of antiplatelet drugs 2-3 days before surgery which did not increase the risk of perioperative bleeding and bleeding-related complications [7]. The 2011 USA edition and 2014 EU edition of guidelines for the treatment of coronary artery reconstruction indicated that patients who intend to undergo CABG should continue to take aspirin preoperatively [8, 9]. In China, the expert consensus on antiplatelet therapy during the perioperative period of coronary artery bypass grafting established in 2016 also pointed out that in principle, it is not recommended to stop aspirin, especially in patients with unstable conditions. However, due to ethnic differences, ecological environment, living environment, and so on, whether or not to stop aspirin before OPCABG is still lacking complete Chinese evidence. This study evaluated the effects of preoperative continuation of aspirin therapy before OPCABG and observed the perioperative performance and physiological indices, to look for evidence of preoperative continuation of aspirin therapy in China.

## 2. Methods

### 2.1. Patients

Between September 2018 and October 2019, a total of 300 patients who received OPCABG for the first time in the hospital were enrolled. All patients were diagnosed with coronary artery disease with severe three-vessel coronary artery disease or left main coronary artery disease. The clinical symptoms included various degrees of chest pain, chest tightness, and restricted mobility. The operation was performed by the same surgical team in the Department of Cardiovascular Surgery, Northern Theater General Hospital. Patients were excluded if they had severe hepatic and renal insufficiency, blood system disease or abnormal coagulation function, allergy to aspirin, or if simultaneous extracorporeal circulation is required.

Blood sampling and inspection are completed by experienced nurses from the Department of Cardiovascular Surgery, Northern Theater General Hospital. The platelet aggregation rate and thromboelastography test are all completed by the Laboratory Department of the Northern Theater General Hospital.

By the table of random numbers, all 300 patients were divided into group A (*n* = 157) and group B (*n* = 143). Group A was subjected to low-molecular-weight heparin 5000 IU subcutaneous injection twice a day and stopped taking aspirin for 5–7 days, while group B accepted heparin as group A plus aspirin 100 mg orally every morning until the day of surgery. A total of 100 patients in the two groups were randomly selected for platelet-related function testing with 48 patients in group A_1_ and 52 patients in group B_1_.

### 2.2. Preoperative Patient Management

After admission, patients were routinely given treatments such as coronary expansion, heart rate control, mild diuresis, and maintenance of electrolyte balance. Patients with a history of hypertension or diabetes were given corresponding antihypertensive and hypoglycemic therapy, and changes in cardiac necrosis indicators such as troponin are monitored. Patients undergoing platelet function testing would be tested for platelet aggregation rate and thromboelastogram on the basis of routine preoperative examinations. Patients with angina pectoris were given nitroglycerin 10 mg sublingually, and those with gradual relief were recorded as one attack of angina pectoris. Patients with no significant relief after coronary drug treatment are diagnosed as acute myocardial infarction, and they will be moved to the cardiovascular surgery intensive care unit as appropriate. A part of them will be implanted with the IABP device to improve myocardial blood supply. All patients were prepared normally before surgery.

### 2.3. Operative Technique

The patient takes the supine position, routinely sterilizes the drape after general anesthesia, takes a median anterior chest incision, and obtains the left internal mammary artery and the corresponding length of the saphenous vein. After the heart was exposed, the location and number of bypass grafts were selected according to the patient's intraoperative coronary artery disease. Intravenous heparin was injected for systemic heparinization. During the operation, the prothrombin activation time (ACT) was maintained >300 s, and the anterior descending artery was fixed with a vascular fixator. Anastomosis of the anterior descending artery with the left internal mammary artery was performed. After the anastomosis was completed, the aorta was partially clamped by the lateral wall clamp, and the proximal end is anastomosed with the great saphenous vein as the graft bridge. Then, the diagonal branch, the obtuse marginal branch, the circumflex distal branch, and the posterior descending branch are fixed with a vascular fixator. According to coronary angiography and intraoperative conditions, the distal of the diseased coronary artery was anastomosed. After transplantation, protamine neutralizing heparin was given, hemostasis was done in the same steps, the pericardium and left thoracic drainage tube were placed during the operation, and all patients returned to the ICU safely. Intensive care personnel will be given corresponding treatment according to the condition. After the hemodynamic index was stable and the spontaneous breathing was completely restored and there was no dyspnea, the tracheal intubation was removed and the condition was stable and transferred to the general ward.

### 2.4. Study Outcomes

During the operation, the blood loss, operation time, and number of graft bridges were recorded in all patients. Patients undergoing platelet function testing were transferred to the ICU after the operation and their condition was stable. Blood was drawn to detect platelet aggregation rate and thromboelastogram. Record the total drainage volume of all patients at 6 h, 24 h after surgery, removal of the surgical drainage tube, postoperative hospital stay, total hospital stay, the number of second thoracotomy, blood transfusion, thoracentesis, and adverse events number. Surgical drainage tubes are generally removed when the postoperative drainage volume is less than 100 ml/24 h, and blood transfusion is given when the intraoperative and postoperative hemoglobin is less than 90 g/L or the hematocrit is less than 25%. When the postoperative drainage volume is greater than 150 ml/h and lasts for 3 h, a second thoracotomy is performed. Antiplatelet drugs were given 6 h after surgery.

### 2.5. Statistical Analysis

All data are statistically analyzed by SPSS 22.0 statistical software. Normally distributed continuous variables are expressed as mean ± standard deviation (SD). Counting data are expressed in number of cases or times (%). Comparison between groups was performed using the *t*-test for normally distributed continuous variables. A paired *t*-test was used for comparison of platelet function related indexes after admission. The chi-square test was used to compare the counting data. Differences were considered significant at *P* < 0.05.

## 3. Results

### 3.1. Group Demographics and Procedural Characteristics

The clinical baseline data of the two groups of patients include the patient's age, gender, BMI, left ventricular ejection fraction (EF value), liver function alanine aminotransferase, history of hypertension, history of diabetes, and history of smoking and drinking history. After statistical analysis of the above clinical data, it was found that it was not statistically significant, as given in Table 1.

### 3.2. Comparison of Preoperative Cardiovascular Events

Statistical analyses revealed that incident rate of preoperative angina in group A was statistically significantly higher than group B (21% vs. 11%, *P* = 0.015). The incidence of new acute myocardial infarction in the two groups (group A vs. group B, 3% vs. 1%, *P* = 0.125), the rate of patients transferred to intensive care unit (4% vs. 1%, *P* = 0.074), and IABP support (3% vs. 1%, *P* = 0.125) between both groups were not statistically significant, as given in Table 2.

### 3.3. Comparison of Intraoperative and Postoperative Observation Indexes

Observe and record intraoperative blood loss, 6 h postoperative drainage volume, 24 h postoperative drainage volume, postoperative total drainage volume, and postoperative drainage tube removal time. The above indicators existing in the two groups had a statistical difference (*P* < 0.05), as given in Table 3 and Figure 1.

Observe and record the operation time, the number of transplanted blood vessels, postoperative hospital stay, total hospital stay, the number of second thoracotomy exploration cases, intraoperative and postoperative red blood cell transfusion, intraoperative and postoperative plasma transfusion, intraoperative and postoperative platelet treatment volume, number of thoracentesis cases, and number of hospital adverse events, and the above indicators existing in the two groups had no statistical difference (*P* > 0.05), as given in Table 3. Adverse events in the hospital include acute cerebral infarction, perioperative myocardial infarction, heart failure, respiratory failure, liver and kidney dysfunction, poor incision healing, and death.

### 3.4. Comparison of Platelet-Related Indexes

On admission, the platelet aggregation rate, thromboelastogram angle, and Ma value of the two groups had no statistical difference (*P* > 0.05), as given in Table 4.

In difference of platelet related indexes after operation, the platelet aggregation rate of the two groups had no statistical significance (*P* > 0.05). The difference of angle and Ma value of the thromboelastogram had no statistical significance (*P* > 0.05), as given in Table 4.

In group A, the platelet aggregation rate, thromboelastogram angle, and Ma value at admission and after operation were compared, and the difference was statistically significant (*P* < 0.05). Among them, the average platelet aggregation rate increased, while the other two averages decreased, as given in Table 5.

Comparing the platelet aggregation rate at admission and postoperation and the angle and Ma value of the thromboelastogram of group B, the difference was found to be statistically significant (*P* < 0.05). Among them, the average platelet aggregation rate increased, and the average of the remaining two items decreased, as given in Table 6.

The angle and Ma values of the thromboelastogram after operation were compared between the two groups. Statistics showed that there was no significant difference in the angle of thromboelastography between the two groups (*P* > 0.05), while the decrease of the Ma value appeared in the two groups. There is a greater decrease in Ma value in the aspirin group after the operation, as given in Table 7 and Figure 2.

## 4. Discussion

For patients with severe coronary artery disease, CABG is still the main method of revascularization, which has been proven to relieve angina and prolong the life expectancy of patients with severe heart disease, especially OPCABG has been an important tool in surgical revascularization [10, 11]. The question of whether to apply antiplatelet drugs before OPCABG has been discussed for many years. Although European and American guidelines recommend that aspirin should be taken orally before surgery until the day of surgery, the practice of relaxing the indications of aspirin has not been widely accepted [12]. Quite a few surgeons believe that stopping aspirin before surgery will increase the number of patients without special anatomy [13]. Nagashima et al. also pointed out that discontinuation of antithrombotic drugs before coronary artery bypass surgery may increase the risk of thromboembolism, but continued use will increase the risk of bleeding [14]. In China, most cardiovascular surgeons also have reservations about the preoperative use of aspirin in patients with coronary artery bypass grafting and still use heparin instead of aspirin before surgery, even though some domestic observational literature has concluded that not stopping aspirin before surgery does not increase OPCABG conclusions on postoperative mortality and risk of intraoperative and postoperative bleeding.

Aspirin is the main therapeutic drug for preventing graft occlusion after coronary artery bypass grafting (CABG) [15–17]. It has been shown to prevent graft failure in patients undergoing coronary artery bypass grafting and ischemic complications such as myocardial infarction and stroke [18]. For patients with coronary heart disease with a long medical history, antiplatelet drugs are usually taken orally before admission, often aspirin, at a dose of 100 mg/day. There is evidence that interruption or discontinuation of low-dose aspirin may cause thrombosis and cause ischemia. The risk of sexual coronary or cerebrovascular events and the risk of death also increase [19]. For patients undergoing OPCABG postoperative graft patency, low blood flow, vasospasm, and vascular endothelial damage may occur during and after the operation, which may promote early graft thrombosis, thereby increasing early or late cardiovascular disease. The risk of events and the use of aspirin can reduce the occurrence of cardiovascular events, and it is recommended to take aspirin immediately before or after surgery to provide related benefits [20].

On the one hand, the positive effect of aspirin on the perioperative period of CABG patients has been continuously proven [21]. On the other hand, there has been controversy about the perioperative risk caused by intraoperative and postoperative bleeding. There are literatures suggesting that in patients undergoing coronary artery surgery, not stopping aspirin before surgery can reduce perioperative myocardial infarction, but it will increase the possibility of bleeding, blood transfusion, and secondary thoracotomy. However, because low-molecular-weight heparin has few side effects and does not increase the risk of intraoperative and postoperative bleeding, low-molecular-weight heparin is still used to replace aspirin [22]. Di Minno et al. [23] pointed out in a review on preoperative treatment of antiplatelet therapy that low-molecular-weight heparin cannot even prevent cardiovascular events. Therefore, compared with low-molecular-weight heparin, aspirin has advantages in preventing cardiovascular events, and replacement therapy alone is not entirely wise.

Whether there was a statistically significant difference in preoperative cardiovascular events between the aspirin group and the aspirin discontinuation group was the first focus of this study. Although there were reports suggesting that low-dose aspirin is associated with a reduction in the probability of severe myocardial infarction throughout the perioperative period, in our study, there was no statistically significant difference in the occurrence of adverse events such as angina or myocardial infarction before surgery [24]. It should be noted that after admission, all patients in the group were given the same treatment plan for coronary expansion, mild diuresis, and maintenance of electrolyte balance, which reduced the occurrence of myocardial ischemia. Therefore, we believe that with adequate medical treatment after admission, the difference between the occurrence of angina pectoris and other adverse events in the two groups before surgery was small.

The second focus of the study is to focus on related indicators such as intraoperative bleeding and postoperative drainage in the two groups of patients. Compared with group A, the aspirin group did increase intraoperative bleeding and postoperative drainage, and the time to remove the surgical drainage tube was also prolonged for a certain period of time [25]. This is also reflected in the actual operation of the operation. The surgeon and assistant can basically accurately judge whether the patient is applying aspirin before the operation in a completely double-blind situation. The main reason is that the incision and wound surface oozes blood [26]. Observing and recording the operation time, the number of graft bridges, the length of hospitalization, blood transfusion, the number of secondary thoracotomy, and the number of related perioperative adverse events in the two groups of patients, the analysis showed that the two groups did not appear on the above indicators, which showed A significant statistical difference. Although the OPCABG intraoperative and postoperative bleeding was more than that of the aspirin group, there was no increase in related complications, and the bleeding risk did not affect the patient's survival rate and was controllable.

Aspirin as a choice for the prevention of graft occlusion and adverse cardiac events after coronary artery bypass graft surgery [27], we want to explore its use on platelet inhibition. Perioperative myocardial infarction is the main cause of morbidity and death after coronary artery bypass grafting, and platelet inhibition has been shown to reduce the incidence of acute bypass occlusion after coronary artery bypass graft surgery [28, 29]. In the study, there was no significant statistical difference in the platelet aggregation rate of the two groups upon admission, but the postoperative test found that the platelet aggregation rate of the two groups showed a certain degree of increase, which may be related to surgery. Although the trend of the two groups was the same, the platelet aggregation rate of the two groups was statistically different after the operation. The platelet aggregation rate of the patients in the aspirin group was significantly lower than that in the discontinuation group. This shows that the preoperative application of aspirin increases the inhibition of platelets in patients during the perioperative period and reduces the risk of adverse cardiovascular events. In addition, there was a statistical difference in the platelet aggregation rate between the two groups in the postoperative and admission levels, which may be related to the body stress caused by the operation.

Thromboelastography is a dynamic depiction of blood clot formation and a sensitive detection method for predicting postoperative thrombotic events in surgical patients. In this study, two indicators, angle and Ma value, were selected to describe platelet function. Although the postoperative indexes of the two groups showed a downward trend compared with the time of admission, there was no statistical difference. At the same time, the statistics of the postoperative and admission indexes in the two groups were different. There was also no significant statistical difference in the angle change between the two groups, but the Ma value showed that the decrease in the aspirin group was greater than that in the aspirin discontinuation group.

Combining the postoperative platelet aggregation rate and the Ma value of the two groups of patients, there are statistical differences in the postoperative decrease in the degree of change compared with the admission. It can be inferred that the aspirin group has more advantages in preventing perioperative cardiovascular events than the aspirin discontinuation group.

## 5. Conclusion

In conclusion, it can be shown that the preoperative application of aspirin has a positive effect on enhancing the platelet inhibitory effect in the early postoperative period among patients with coronary heart diseases, and furthermore, it would increase the risk of intraoperative and postoperative hemorrhage; nonetheless, this risk is controllable and has not increased the occurrence of adverse events such as cardiovascular events, and at the same time, it has enhanced the inhibiting effect on platelets.

## Figures and Tables

**Figure 1:** Intraoperative and postoperative bleeding statistics.

**Figure 2:** Chart of the amplitude of change in Ma value.

**Table 1:** Statistical table of patients' clinical data comparison between the ceasing group and coutilization group.

	Group A (*n* = 157)	Group B (*n* = 143)	*P* value
Age (year)	61.7 ± 7.89	62.42 ± 7.68	0.519
Gender (male)	118 (75%)	113 (79%)	0.541
BMI (kg/m^2^)	24.9 ± 3.43	25.21 ± 3.30	0.724
Hypertension (*n*)	110 (70%)	96 (67%)	0.658
Diabetes (*n*)	55 (35%)	50 (35%)	0.984
LVEF	0.55 ± 0.04	0.55 ± 0.04	0.710
Liver function (ALT U/L)	27.87 ± 14.28	26.37 ± 17.93	0.503
Smoking (*n*)	89 (57%)	89 (62%)	0.522
Drinking (*n*)	26 (16%)	34 (24%)	0.221

**Table 2:** Statistical table of preoperative cardiovascular events in the ceasing group and coutilization group.

	Group A (*n* = 157)	Group B (*n* = 143)	*P* value
Preoperative angina (*n*/%)	34 (21%)	16 (11%)	0.015^*∗*^
Acute myocardial infarction preoperatively (*n*/%)	5 (3%)	1 (1%)	0.125
Preoperative IABP support (*n*/%)	5 (3%)	1 (1%)	0.125
Transferred to intensive care unit (*n*/%)	6 (4%)	1 (1%)	0.074

Significant difference, ^*∗*^*P* < 0.05.

**Table 3:** Statistical table of intraoperative and postoperative hemorrhage and cardiovascular events in the ceasing group and coutilization group disscussion.

	Group A (*n* = 157)	Group B (*n* = 143)	*P* value
Intraoperative blood loss (ml)	304.54 ± 68.69	361.67 ± 72.94	≤0.001^*∗*^
Time of operation (min)	239.59 ± 44.10	236.50 ± 32.43	0.586
Grafted vessels	3.35 ± 0.68	3.27 ± 0.59	0.128
6 hours postoperative drainage (ml)	210.67 ± 62.51	275.18 ± 81.02	≤0.001^*∗*^
24 hours postoperative drainage (ml)	460.17 ± 113.66	577.44 ± 163.15	≤0.001^*∗*^
Total drainage volume (ml)	1382.90 ± 621.05	1667.98 ± 722.02	0.003^*∗*^
Time to remove the drainage tube (h)	121.22 ± 43.74	136.56 ± 57.34	0.032^*∗*^
Hospital stays after surgery (day)	10.62 ± 4.02	11.03 ± 3.72	0.630
Hospital stays (day)	23.71 ± 7.29	23.54 ± 7.32	0.864
Secondary thoracotomy (*n*)	0 (0%)	2 (1%)	0.155
RBC transfusion (U)	0.30 ± 0.86	0.51 ± 1.12	0.138
Infusion plasma (ml)	35.17 ± 127.01	56.07 ± 161.95	0.303
Platelet transfusion	0.01 ± 0.09	0.04 ± 0.19	0.167
Thorax puncture (*n*)	13 (8%)	9 (9%)	0.507
Adverse event (*n*)	6 (4%)	9 (6%)	0.607

**Table 4:** Statistical table of platelet relevant indicators in the ceasing group and coutilization group.

	Group A (*n* = 48)	Group B (*n* = 52)	*P* value
Platelet aggregation rate (%)	32.71 ± 27.02	24.68 ± 17.21	0.114
Angle (°)	65.74 ± 6.32	67.09 ± 5.99	0.553
Ma (mm)	60.86 ± 6.71	63.59 ± 6.75	0.074
Postoperative platelet aggregation rate (%)	58.38 ± 28.15	35.36 ± 26.84	≤0.001^*∗*^
Postoperative angle (°)	60.51 ± 8.33	60.80 ± 6.70	0.912
Postoperative Ma (mm)	57.90 ± 6.60	58.86 ± 6.07	0.501

**Table 5:** Statistical table of preoperative and postoperative platelet relevant indicator comparison in the ceasing group.

	On admission	Postoperative	*P* value
Platelet aggregation rate (%)	32.71 ± 27.02	58.38 ± 28.15	0.001^*∗*^
Angle (°)	65.74 ± 6.32	60.51 ± 8.33	0.029^*∗*^
Ma (mm)	60.86 ± 6.71	57.90 ± 6.60	≤0.001^*∗*^

**Table 6:** Statistical table of preoperative and postoperative platelet relevant indicator comparison in the coutilization group.

	On admission	Postoperative	*P* value
Platelet aggregation rate (%)	24.68 ± 17.21	35.36 ± 26.84	0.012^*∗*^
Angle (°)	67.09 ± 5.99	60.80 ± 6.70	0.009^*∗*^
Ma (mm)	63.59 ± 6.75	58.86 ± 6.07	≤0.001^*∗*^

**Table 7:** Statistical table of thromboelastography rangeability after admission in the ceasing group and coutilization group.

	Group A_1_ (*n* = 48)	Group B_1_ (*n* = 52)	*P* value
Postoperative angle on admission, angle (°)	5.24 ± 7.99	6.29 ± 8.56	0.718
Postoperative Ma on admission, Ma (mm)	2.64 ± 4.32	5.04 ± 5.72	0.037^*∗*^

## Data Availability

The data used to support the findings of this study are available from the corresponding author upon request.
